# Clinical Efficacy of CT-Guided Continuous Catheterization Drainage for Spinal Tuberculosis with Large Abscesses

**DOI:** 10.1155/2022/2402048

**Published:** 2022-01-27

**Authors:** Shengxun Zhang, Dengfeng Li, Liang Liang, Zhen Tian, Zeyu Sun, Yuekui Jian

**Affiliations:** ^1^Guizhou University Medical College, Guiyang City, Guizhou Province, China; ^2^Orthopedics Department, Guizhou Provincial People's Hospital, Guiyang City, Guizhou Province, China

## Abstract

**Objective:**

This study aimed to determine the efficacy of computed tomography (CT)-guided local catheterization for the treatment of spinal tuberculosis (TB) with abscess.

**Methods:**

Clinical data from 22 cases of lumbar TB with abscess receiving treatments from July 2015 to January 2021 were analyzed. Some patients (*n* = 11) underwent pure surgery (control group) and the others (*n* = 11) received CT-guided catheterization drainage. The operation and hospitalization time, erythrocyte sedimentation rate (ESR), visual analog scale (VAS), ASIA damage grade, and C-reactive protein (CRP) levels of both groups were compared.

**Results:**

The operation time, intraoperative blood loss, and hospital stay of the observation group were significantly less than those of the control group (*P* < 0.05). As the differences in preoperative ESR, CRP, and VAS scores between both groups did not reach significance (*P* > 0.05), after treatments, the observation group had a lower level of ESR and CRP (*P* < 0.05); the postoperative VAS scores of the two groups decreased (*P* > 0.05). Before treatment, the control group comprised 2 cases of ASIA grade A, 1 case of B, 6 cases of C, and 2 cases of D with 3 patients having dyskinesia. After surgery, the motor function of the patients was improved, and there were 3 cases of ASIA D and 8 cases of E. Meanwhile, the preoperative observation group consisted of 9 cases of ASIA D and 2 cases of E. Due to CT-guided catheterization, all patients achieved clinical healing (ASIA E) when the lesions were significantly alleviated, and symptoms such as low back pain and lower extremity pain disappeared.

**Conclusion:**

CT-guided percutaneous catheter drainage for continuous administration of drugs is effective treatment for spinal TB with abscess, when shortening the operation and hospitalization time and reducing intraoperative blood loss and erythrocyte sedimentation rate. It is worthy of popularization and application.

## 1. Introduction

Following global COVID-19 epidemic, the numbers of new tuberculosis (TB) patients in 2020 kept increasing month by month. Osteoarticular TB is one of the symptoms of systemic TB [1], whilst bone TB makes up 10% of extrapulmonary cases, and 50% of bone TB occurs in the spine [2]. Lumbar TB and thoracic TB are the most common form of spinal TB; without any typical symptoms in the early stage, patients spinal TB are usually diagnosed at an advanced stage when having large spinal tuberculous abscesses [3]. Abscesses are first present in front of vertebral body or beneath vertebral periosteum; as the condition progresses, gravitation abscess lifts up the periosteum of spinal vertebrae and adjacent vertebrae to form a large paravertebral abscess, which causes localized pain and mass and even paraplegia due to compression of the spinal cord by the accumulation of pus in the spinal canal [4]. However, the efficacy of conservative or surgical management is not ideal [5]. Clinically, continuous administration of anti-TB drugs via computed tomography (CT)-guided percutaneous catheterization and drainage lavage are widely applied to practice and have great therapeutic advantages. This study aimed to determine the efficacy of CT-guided local catheterization for the treatment of spinal TB with abscess.

## 2. Materials and Methods

### 2.1. Patient Information

From July 2015 to January 2021, 22 cases of lumbar TB diagnosed in Guizhou Provincial People's Hospital were enrolled in the present study, and all participants met the inclusion criteria [6] and had large abscesses without open TB. These patients were divided into the control group and observation group (*n* = 11), including 8 cases of thoracic TB, 12 cases of lumbar TB, and 2 cases of left joint TB. There was no significant difference in patient's data (*P* > 0.05) (Table 1).

## 3. Methods

### 3.1. Preoperative Preparation

Like other operations, patients received routine inspections before surgery.

### 3.2. Operating Steps

In the control group, different surgical approaches were used according to the location and existence of spinal instability, including anterior, posterior, and lateral approaches. The operation lasted an average of 6 hours and stayed in bed for 6 weeks [4]. As for the observation group, patients received puncture angiography under local infiltration anesthesia with aseptic operation and draping. The 18G trocar needle was inserted into abscesses under DynaCT through percutaneous puncture for localization. When the drawn liquid was yellow pus, the position was confirmed by angiography, and a 0.035 inch guide wire then was inserted with a 6F dilator used to expand the puncture tract. Then, the expander and 8.5 F multibranch drainage catheter were coaxially placed into the abscess and fixed. The doctor then resuscitated the patient and returned to the ward. Some sacroiliac joints require internal fixation with screws.

### 3.3. Postoperative Treatment

Patients were commended to assure adequate bed rest, sufficient nutrition, and physical exercises and to avoid cold and strenuous weight-bearing activities at the waist. 0.3 g isoniazid and 0.5 rifamycin were used once a day for 2 months for irrigation of the abscess cavity everyday with the drainage tube to keep clean. The dressing should be changed every 2-3 days with disinfection. After discharge, patients kept receiving oral anti-TB medicine for at least 18 months: ethambutol 0.75 g/day once a day, rifampicin 0.45 g/day once a day, pyrazinamide 0.75 g/day twice a day in the morning, and isoniazid 0.3 g/day once a day. Taking into account the side effects of tuberculosis drugs on the liver and kidneys, liver and kidney function should be monitored, and relevant indicators should be reviewed monthly during the oral period.

### 3.4. Follow-Up Indicators

After treatments, the relevant indicators of the two groups were compared. The clinical evaluation of the visual analog scale (VAS) is divided into five grades: A, B, C, D, and E [7]. According to the American Spinal Injury Association (ASIA) Classification, spinal cord injury was classified as A: complete damage, B: incomplete damage with sensation, C: incomplete damage with preserved motor function, D: moderate damage, and E: normal sensation and motor function.

### 3.5. Statistical Analysis

All data were processed by SPSS software. Measurement data were presented as mean ± standard error (*X* ± *s*), and qualitative data were represented as (*n*)%. The *t*-test and *χ*^2^ test were used for analysis. *P* < 0.05 indicates statistical significance.

## 4. Results

### 4.1. Comparison of Preoperative and Postoperative Imaging in Individual Patients

Imaging examination showed that the preoperative paravertebral abscess was large, 76.95 ± 12.63 mm in diameter, with obstructive organ function. After percutaneous catheterization and drug treatment, the abscess decreased significantly, as shown in Figure 1.

### 4.2. Comparison of Relevant Indicators of Patients

The operation time (1.68 ± 0.17 h), intraoperative blood loss (618.36 ± 183.37 mL), and hospitalization time (12.55 ± 1.19 d) of the observation group were significantly lower than those of the control group (9.32 ± 0.70 h, 1350.18 ± 241.20 mL, and 15.64 ± 1.89 d) (*P* < 0.05), as given in Table 2.

### 4.3. Comparison of Other Relevant Indicators between Both Groups

Comparing the patient's data (Table 3), the preoperative ESR, CRP levels, and VAS scores between the two groups were not significantly different (*P* > 0.05). After treatments, the ESR and CRP levels of the two groups were significantly reduced, and the observation group had the lower levels (*P* < 0.05). ESR and CRP returned to normal level one month after catheterization drainage, and their levels in the control group recovered slowly and did not reach normal levels. While the VAS score upon treatments decreased in both groups, there was no significant difference in the postoperative VAS score (*P* > 0.05).

### 4.4. ASIA Grades in the Two Groups

Before treatment, according to ASIA classification, the numbers of cases with ASIA A, B, C, and D were 2, 1, 6, and 2, as 3 patients exhibited various degrees of dyskinesia. After surgery, the motor function of the patients was improved, and there were 3 cases of ASIA D and 8 cases of E. Meanwhile, the preoperative observation group consisted of 9 cases of ASIA D and 2 cases of E. Due to drug treatment via CT-guided catheterization, all patients achieved clinical healing (ASIA E) when the lesions were significantly alleviated, and low back pain and lower extremity pain disappeared (Table 4).

## 5. Discussion

Spinal TB is most frequently located in lumbar vertebrae, followed by thoracic vertebrae, which induces injuries and eventually compresses spinal cord and causes paraplegia in severe cases [8]. CT is a minimally invasive technique reducing postoperative pain and resulting in fast recovery; it clearly displays the structures with very small density so that the vertebral body and nearby anatomical structures and pathological structures can be observed through it [7]. For spinal TB, CT-guided percutaneous catheterization is confirmed to accurately puncture into the lesion and relieve the patient's pain, safely and reliably [4, 6, 9]. Besides, local chemotherapy is reported to greatly increase the concentration of the drug with greater efficacy [10], so it has a greater therapeutic value.

The data of our study demonstrate that CT-guided percutaneous catheterization exhibits greater effectiveness in the treatment of spinal TB with large abscesses than conventional approaches, consistent with the conclusion drawn by Pombo et al. [11]. A study in 2003 has already indicated that continuous administration of local chemotherapy and drainage in the treatment for 15 cases of spine TB successfully enabled ESR to return to the normal level [12]. Additionally, Mengqi et al. reported that efficacy of continuous local administration to abscess absorption reached as high as 84% [13]. Wu et al. also noted that local chemotherapy has lower recurrence rate and greater effectiveness [4]. In a study of Zou et al., 16 patients underwent two-stage CT-guided percutaneous abscess drainage and posterior debridement, decompression, intervertebral fusion, and device treatment; the neurological deficits were recovered to varying degrees with significantly improved patients' life quality [14].

With the increasing drug resistance of mycobacterium TB, CT-guided percutaneous catheter drainage for continuous administration of drugs effectively improves spinal TB with huge abscesses, not only reducing the operation time, pain, and blood loss but also achieving complete removal of the lesions with great efficacy. Collectively, the therapeutic regimen in this study has a great curative effect on spinal TB with large abscesses and has an important application value.

## Figures and Tables

**Figure 1:** Comparison of preoperative and postoperative imaging. (a) The coronal plane imaging of preoperative paravertebral abscess. (b) The coronal plane imaging of the paravertebral abscess after the operation. (c) The sagittal plane of preoperative paravertebral abscess before surgery. (d) The sagittal plane imaging of postoperative paravertebral abscess after surgery.

**Table 1:** Comparison of general information of the two groups (*x* ± *s*).

Group	Average age (years)	Gender (*n*)	
		Male	Female
Control group (*n* = 11)	44.13 ± 4.96	6	5
Observation group (*n* = 11)	43.91 ± 4.97	5	6
*t*/*χ*^2^	0.090	0.182	
*P* value	0.929	0.670	

**Table 2:** Comparison of general data between the two groups (*x* ± *s*).

Group	Operation time (h)	Intraoperative blood loss (mL)	Hospitalization time (d)
Observation group (*n* = 11)	1.68 ± 0.17	618.36 ± 183.37	12.55 ± 1.19
Control group (*n* = 11)	9.32 ± 0.70	1350.18 ± 241.20	15.64 ± 1.89
*t*	35.182	8.011	4.589
*P*	<0.001	<0.001	<0.001

**Table 3:** Comparison of various indexes of the two groups before and after surgery (*x* ± *s*).

Group	ESR(mm/h)		CRP(mg/L)		VAS (minutes)	
	Before surgery	After surgery	Before surgery	After surgery	Before surgery	After surgery
Observation group (*n* = 11)	52.00 ± 11.80	9.18 ± 1.20^*∗*^	47.97 ± 8.32	5.79 ± 1.35^*∗*^	4.82 ± 0.26	0.82 ± 0.23^*∗*^
Control group (*n* = 11)	53.36 ± 6.20	25.82 ± 4.35^*∗*^	46.13 ± 7.09	21.88 ± 4.26^*∗*^	4.82 ± 0.38	1.00 ± 0.27^*∗*^
*t*	0.338	12.231	0.558	11.942	<0.001	1.683
*P*	0.739	<0.001	0.583	<0.001	>0.999	0.108

*Note.* ^*∗*^ vs. before operation, *P* < 0.05.

**Table 4:** Comparison of ASIA grade before and after operation between the two groups (*n*).

Group	Preoperative ASIA level					Postoperative ASIA level				
	A	B	C	D	E	A	B	C	D	E
Observation group (*n* = 11)	0	0	0	9	2	0	0	0	0	11
Control group (*n* = 11)	2	1	6	2	0	0	0	0	3	8

## Data Availability

The data used to support the findings of this study are available from the corresponding author upon request.
